# Correlation between Sleep Time, Sleep Quality, and Emotional and Cognitive Function in the Elderly

**DOI:** 10.1155/2022/9709536

**Published:** 2022-05-14

**Authors:** Heng Liao, Sha Liao, Yu-jiao Gao, Jing-ping Mu, Xi Wang, De-sen Chen

**Affiliations:** Sleep Psychosomatic Medicine Center, Taihe Hospital of Shiyan City, Hubei University of Medicine, 442000, China

## Abstract

**Background:**

To explore the relationship between sleep time, sleep quality, and emotional and cognitive function in the elderly.

**Methods:**

A total of 150 elderly patients over 65 years old who were admitted to our hospital from February 2019 to April 2021 were divided into a normal cognitive function group (Mini-Mental State Examination (MMSE) score: illiteracy, >17; primary school, >20; and middle school and above, >24; *N* = 86) and cognitive impairment group (MMSE score: illiteracy, ≤17; primary school, ≤20; and middle school or above, ≤24; *N* = 64). The sleep quality was evaluated by the Pittsburgh Sleep Quality Index (PSQI), and anxiety and depression were evaluated by Hamilton anxiety scale (HAMA) and Hamilton depression scale (HAMD), respectively. The cognitive function between the two groups was compared via the Montreal Cognitive Assessment (MoCA) score, visual spatial execution, and attention. Pearson correlation analysis was used to analyze the correlation between sleep quality, sleep time, and emotional and cognitive function.

**Results:**

In the comparison of sleep quality between the two groups, the total score of PSQI, sleep quality, falling asleep time, sleep time, and sleep efficiency of patients with cognitive impairment were higher than those of patients with normal cognitive function (*P* < 0.05). There was no significant difference in the scores of hypnotic use and daytime dysfunction between the two groups, but the scores of nocturnal sleep disorders and ESS in the cognitive impairment group were significantly higher than those in the normal group (*P* > 0.05). Compared between the two groups, the MoCA score, visual spatial execution, and attention in the cognitive impairment group were significantly lower than those in the normal group, and the difference was statistically significant (*P* < 0.05). The delayed recall in the cognitive impairment group was significantly higher than that in the control group (*P* < 0.05). There was no significant difference in orientation, naming, language, and abstract ability between the two groups (*P* > 0.05). The scores of HAMA and HAMD in the cognitive impairment group were significantly higher than those in the normal group. Pearson correlation analysis was used to analyze the correlation between sleep therapy, sleep time, and the score of cognitive scale. The results showed that PSQI was negatively correlated with MoCA and MMSE, and ESS was negatively correlated with MoCA and MMSE. Pearson correlation analysis results indicated that PSQI was positively correlated with HAMA and HAMD, while ESS was negatively correlated with HAMA and HAMD.

**Conclusion:**

The sleep quality and sleep time of elderly patients are positively correlated with their cognitive function. The worse the sleep quality is, the worse their cognitive function is and the more serious their anxiety and depression are. In the course of clinical therapeutics, more attention should be paid to the sleep quality of elderly.

## 1. Introduction

Cognitive function is an advanced neural activity function of the human brain functional cortex to obtain, convert, and conduct external objective information, which is mainly composed of memory, calculation, visual space ability, execution ability, and other fields [1–3]. The main symptoms of cognitive dysfunction are decline in memory and vision, executive dysfunction, and dementia, while dementia is the outcome of severe cognitive impairment, which seriously impairs the life quality of patients and increases the burden of society and family [4, 5]. The number of people with cognitive impairment and dementia is increasing rapidly at a rate of 300,000 per year [6]. Recent epidemiological data indicate that the prevalence of dementia in the elderly in China is 3%-5% [7, 8], and the prevalence rate of mild cognitive impairment is 20% [9, 10]. Cognitive function is in association with many factors, such as social demographic characteristics, lifestyle, physical function, disease, and psychology [10]. Notably, the relationship between sleep quality and cognitive function has attracted much attention in recent years. Some studies have reported that the decrease in sleep quality is closely related to the increased risk of cognitive decline [11]. Sleep disorders mainly include insomnia, sleep apnea syndrome, restless leg syndrome, periodic limb movement disorders, biorhythmic sleep disorders, secondary insomnia, subjective insomnia, and short sleep [12, 13]. Sleep disorders can promote mental, neurological, and subhealth symptoms, provoke a variety of complications, affect the normal life of patients, and endanger their health. With the aging of the population and the sharp increase in various adverse social and environmental factors, the proportion of people with sleep disorders in China has reached 9%, and it has even been reported that the proportion is as high as 41% over the age of 60 [14]. There is a close relationship between sleep disorder and cognitive function. In our current study, this research focuses on 72 elderly patients aged ≥63 treated in our hospital from February 2019 to April 2021, which are reported as follows.

## 2. Cases and Methods

### 2.1. General Clinical Information

A total of 150 elderly patients over 65 years old who were admitted to our hospital from February 2019 to April 2021 were divided into a normal cognitive function group (MMSE score: illiteracy, >17; primary school, >20; and middle school and above, >24; nasty 86) and cognitive impairment group (MMSE score: illiteracy, ≤17; primary school, ≤20; and middle school or above, ≤24; *N* = 64). In the normal cognitive function group, the age was from 65 to 80 years, with an average age of 75.34 ± 6.61 years, including 20 males and 16 females, and in the cognitive impairment group, the age was from 66 to 82 years, with an average age of 76.87 ± 7.08 years, including 18 males and 18 females. There was no statistical significance in the general data of the two groups. This study was approved by the Medical Ethics Association of our hospital, and all patients signed informed consent.

The inclusion criteria were as follows: (1) ≥65 years old and able to complete various scales and examinations; (2) patients with normal cognitive function had no cognitive, language, and intellectual impairment and had basic reading and writing ability; (3) MMSE scores of patients with cognitive impairment did not reach the standard of dementia; and (4) activities of daily living were not affected, and they could complete daily life and diet independently and ADL scale (activities of daily living).

Exclusion criteria were as follows: (1) patients with severe heart, liver, and renal insufficiency, malignant tumors, and other diseases; (2) exclusion of severe emotional disorders such as anxiety and depression or mild cognitive impairment caused by medication, which affect the accuracy of cognitive assessment results; (3) exclusion of mild cognitive impairment caused by other diseases (such as PD, encephalitis, hypothyroidism, and other systemic diseases); (4) ruling out other diseases that affect sleep, such as nocturnal urination, drunkenness, asthma, and chronic pain; and (5) excluding those who suffered from serious medical diseases and heart, liver, lung, and kidney basic diseases and cannot cooperate with the completion of the study.

### 2.2. Research Methods

In this study, general personal information was collected from all participants, including age, sex, height, weight, occupation, education level, and current medical history, past history, personal history, and family history. Then, we improved the basic items of blood sampling: blood routine, liver and kidney function, biochemistry, blood lipids, and so on. Improve blood sampling (thyroid function, vitamin B12, folic acid, homozygous hemispheric acid HIV antibody, and syphilis infectious examination) and head magnetic resonance plain scan (if the patient cannot cooperate, head CT is recommended).

Furthermore, in this study, all the participants were assessed by trained cognitive and psychological scale evaluators, and the correlation between sleep time, sleep quality, and emotional and cognitive function in elderly patients was analyzed by Pearson correlation analysis.

### 2.3. Observation Index

#### 2.3.1. Mini-Mental State Examination (MMSE) Score

The MMSE scale [15] is short and feasible. It has general sensitivity and specificity in distinguishing normal elderly and MCI patients, which plays an important role in evaluating and monitoring the moderate and severe dementia in patients diagnosed with dementia. MMSE is widely used in clinic and often functions as a cognitive screening tool in clinic. The questions in the table included orientation, immediate recall, delayed recall, computational power, attention, visual space, language, and other cognitive domains, with a total score of 30.

#### 2.3.2. Montreal Cognitive Assessment (MoCA) Score

The Montreal Cognitive Assessment scale [16] (MoCA), developed by Professor Nasreddine in 2004, was an assessment tool for rapid screening of mild cognitive impairment (MCI). The assessed cognitive areas included attention and concentration, executive function, memory, language, visual structure skills, abstract thinking, calculation, and orientation. The total score of the scale is 30, and the test results show that the normal value is ≥26.

#### 2.3.3. PSQI Score

Pittsburgh Sleep Quality Index (PSQI) scale [17], made by the University of Pittsburgh in 1980, is mainly used to evaluate the sleep quality of patients with sleep and mental disorders. PSQI is a subjective sleep assessment scale and is widely used in clinic. PSQI includes seven subitems: sleep quality, time to fall asleep, sleep efficiency, sleep disorders, hypnotic use, and daytime dysfunction. Each subitem has 3 points, and the score > 7 can be regarded as the existence of sleep disorder. The higher the score, the more serious the sleep disorder.

#### 2.3.4. ESS Score

The ESS scale [18] is mainly designed for daytime sleep disorders in recent months and is used to evaluate whether excessive drowsiness exists during the day. The score > 6 indicates the existence of daytime drowsiness, >11 indicates the existence of excessive drowsiness, and >16 indicates the existence of dangerous drowsiness.

#### 2.3.5. HAMA Score

The Hamilton anxiety scale (HAMA) [19] was compiled in 1959 and has been widely used in clinic. In principle, the scale needs to be assessed by two professionals, via the way of conversation. Due to the limitation of human resources, we evaluate the patients by one person. The version used in the study was the HAMA14 version. <7 indicated that there was no anxiety, ≥14 indicated that there must be anxiety, ≥21 considered that there was obvious anxiety, and ≥29 indicated that there was serious anxiety.

#### 2.3.6. Life Quality Scale

In the Hamilton depression scale (HAMD) [20], the basic description is the same as the HAMA scale. The first scale is used as the most basic tool to evaluate the efficacy of antidepressants in the field of antidepressant therapy. We use the HAMD 17 version. Scores < 7 indicate that there is no depression, scores ≥ 17 are considered mild to moderate depression, and scores ≥ 24 may be considered severe depression.

### 2.4. Statistical Analysis

SPSS21.0 statistical software was employed; before statistical analysis, the measurement data were tested by normal distribution and variance homogeneity analysis to meet the requirements of normal distribution or approximate normal distribution, expressed as $\bar{x}\pm \text{s}$. The *t*-test was used to compare the two groups. *N* (%) was used as an example to represent the counting data. The *χ*^2^ test and Pearson correlation analysis were used to analyze the correlation between sleep timing, sleep quality, and emotional and cognitive function in the elderly.

## 3. Results

### 3.1. Comparison of Sleep Quality between the Two Groups

The total score of PSQI, sleep quality, falling asleep time, sleep time, and sleep efficiency in the cognitive impairment group were higher than those in the normal cognitive function group (*P* < 0.05). The total score of sleep quality, sleep quality, sleep time, and sleep efficiency in the cognitive impairment group were significantly higher than those in the normal cognitive function group (*P* < 0.05). All the results are shown in Table 1.

### 3.2. Comparison of Sleeping Subitem Scores between the Two Groups

There was no significant difference in the scores of hypnotic use and daytime dysfunction between the two groups, but the scores of nocturnal sleep disorders and ESS in the cognitive impairment group were significantly higher than those in the normal cognitive function group (*P* > 0.05). The results are shown in Table 2.

### 3.3. Comparison of Cognitive Function between the Two Groups

Compared between the two groups, the MoCA score, visual spatial execution, and attention in the cognitive impairment group were significantly lower than those in the normal cognitive function group, and the difference was statistically significant (*P* < 0.05). The delayed recall in the cognitive impairment group was significantly higher than that in the control group (*P* < 0.05). There was no significant difference in orientation, naming, language, and abstract ability between the two groups (*P* > 0.05). The results are shown in Tables 3 and 4.

### 3.4. Comparison of Anxiety and Depression Scores between the Two Groups

The scores of HAMA and HAMD in the cognitive impairment group were significantly higher than those in the normal cognitive function group. The results are shown in Table 5.

### 3.5. Correlation between Sleep Quality, Sleep Time, and Cognitive Scale Scores

Pearson correlation analysis was performed to analyze the correlation between sleep therapy, sleep time, and the score of cognitive scale, and the results indicated that there was a negative correlation between PSQI and MoCA or MMSE (*r* = −0.487, -0.634, *P* < 0.05). Moreover, there was a negative correlation between ESS and MoCA or MMSE(*r* = −0.517, -0.532, *P* < 0.05). The results are shown in Table 6.

### 3.6. Correlation between Sleep Quality, Sleep Time, and Emotional Score

Pearson correlation analysis was conducted to analyze the correlation between sleep therapy, sleep time, and emotional score. The results indicated that there was a positive correlation between PSQI and HAMA or HAMD (*r* = 0.237, 0.218, *P* < 0.05). Moreover, there was a negative correlation between ESS and HAMA or HAMD (*r* = −0.416, -0.387, *P* < 0.05). The results are shown in Table 7.

## 4. Discussion

Sleep is an important physiological process involved in various body function recoveries. With the increase in age, there are remarkable qualitative and quantitative changes in sleep. Some studies have found that [21, 22] the mortality rate increases with age, and the mortality rate of patients with cognitive impairment is also higher [22]. Notably, sleep disorders and cognitive disorders are common in the elderly. There is growing evidence of a potential link between sleep and cognitive function. Changes in sleep patterns tend to occur with age, including decreased total sleep time and efficiency, increased sleep fragmentation, more difficulty to fall asleep, and less time for rapid eye movement (REM) sleep and slow wave sleep.

Studies have revealed that [23–25] REM sleep disorder is often accompanied by Louis bodies, suggesting changes in the structure of the brainstem, although there is no anatomical evidence. There are a variety of research results on sleep disorders in the elderly, but they all suggest that there is a certain relationship between poor sleep quality and cognitive impairment. Four prospective studies used subjective sleep quality assessment tools to evaluate sleep quality, one of which showed a correlation between poor sleep quality and cognitive decline [23]. In addition, other results show that poor sleep quality increases the risk of cognitive impairment and dementia. The rate of cognitive decline was two to four times higher in people with sleep disorders than in those without sleep disorders [24–26]. However, two prospective studies [27, 28] followed up for 2 years or 8 years indicated that there was no significant association between poor sleep quality and decreased cognitive function. Some scholars have pointed out that the mechanism of the effect of sleep quality on cognitive function is as follows: (1) abnormal clearance of *β*-amyloid protein: sleep participation includes physiological processes such as the recovery of brain function and the clearance of brain metabolites, including *β*-amyloid protein (A*β*); (2) inflammation: lack of sleep promotes inflammation, which accelerates the process of neurodegeneration in key areas or the hippocampus related to learning and memory, which brings about the decline of cognitive function; (3) abnormal function and melatonin secretion of the suprachiasmatic nucleus (SCN) in the anterior hypothalamus: SCN is the most important endogenous pacemaker in the sleep awakening cycle; the pineal gland secretes melatonin after being stimulated by SCN, and melatonin can promote sleep and protect nerves; and (4) sleep disorders such as insomnia and sleep deprivation can damage the cAMP and GABA signal pathways of neurons and affect the synaptic plasticity of neurons. Our present study focused on the elderly over 65 years old, and the results indicated that the total score of PSQI, sleep quality, falling asleep time, sleep time, and sleep efficiency in the cognitive impairment group were higher than those in the normal cognitive function group. The score of nocturnal sleep disorder in the cognitive impairment group was significantly higher than that in the normal cognitive function group, and the ESS score in the cognitive impairment group was significantly higher than that in the normal cognitive function group. Moreover, the MoCA score, visual spatial execution, and attention in the cognitive impairment group were significantly lower than those in the normal cognitive function group, while the delayed recall in the cognitive impairment group was significantly higher than that in the control group. In order to further clarify the correlation between sleep quality and cognitive function in elderly patients, this study was analyzed by Pearson correlation analysis. The results showed that PSQI and ESS were negatively correlated with MoCA and MMSE. This showed that the sleep quality of elderly patients would exert a negative impact on their cognitive function. Jiang et al. [29] took 2932 women ≥ 65 years old as subjects, counted their sleep time by self-reported daily TST, and evaluated their cognitive function by the global cognitive function test, and no correlation was found between them. Mahendran et al. [30] utilized PSQI and MoCA to evaluate sleep quality and cognitive function in 88 patients with chronic obstructive pulmonary disease (COPD), and the results found that there was a negative correlation between sleep efficiency and delayed recall, which was consistent with our study. This study also established that patients with COPD have more impairment of executive function, delayed memory, language, and abstract ability, which may be linked to the disease characteristics of the study population and the cognitive function assessment scale evaluated by MoCA. At present, there are several possible neurobiological evidences to explain the relationship between long sleep time and cognitive impairment. First, studies have shown that long periods of sleep can accelerate frontotemporal gray matter atrophy in older people, which may damage memory. Long-term sleep may reflect sleep disorders and cognitive impairment related to circadian rhythm disorders, which is basically consistent with the conclusions of our study.

A meta-analysis [31] shows that anxiety increases the risk of cognitive impairment and Alzheimer's disease, which is more significant in older people, and anxiety may be a precursor of cognitive impairment. A cross-sectional study [32] presents that severe anxiety can promote distraction and cognitive impairment, and the potential mechanisms include hypercortisolism, cardiovascular disease, low level of inflammation, BDNF inhibition, and cognitive reserve. Furthermore, anxiety can contribute to an increase in cortisol secretion [33]. The research reported that people with high cortisol had lower scores on neuropsychological tests than those in the normal control group, because cortisol stimulates adrenocortical hormone receptors in the medial temporal lobe, leading to hippocampal atrophy [32]. In animal models, high cortisol can also give rise of A*β* deposition and tau protein deposition. The above two processes will lead to the decline of cognitive function. Some studies have found that anxiety is related to coronary heart disease and stroke. Stress caused by anxiety can trigger physiological responses, such as increased heart rate, elevated blood pressure, vasoconstriction, and platelet activity, which are associated with heart-related vascular disease and can lead to vascular dementia. Low levels of inflammation, such as the increase in IL-6 and TNF, are related to anxiety, and the increase in these inflammatory factors will adversely affect cognitive function. Anxiety is also related to BDNF, while BDNF is involved in synaptic plasticity, learning and memory, and nerve repair. The present study demonstrated that BDNF levels decreased in both mild cognitive impairment and Alzheimer's disease. Another explanation may be that a reduction in cognitive reserve increases the risk of dementia and that anxiety has a persistent course through life and is accompanied by avoidance behaviors, which may be due to a reduction in mental and social stimulation leading to a reduction in cognitive reserve [33]. The results of this study showed that the scores of HAMA and HAMD in the cognitive impairment group were significantly higher than those in the normal cognitive function group. PSQI was positively correlated with HAMA and HAMD, while ESS was negatively correlated with HAMA and HAMD. Thus, it can be acknowledged that poor sleep quality can bring about the aggravation of anxiety and depression, while the accumulation of bad emotions will further aggravate the impairment of cognitive function in a manner of negative feedback.

Moreover, at present, there are some limitations in the research on the relationship between sleep quality and cognitive function, which are shown in the following aspects: (1) considering the many factors associated with cognitive function, including age, gender, education level, blood lipids, disease status, and medication use, the accuracy of the results remains limited, although by adjusting for confounding factors. (2) The sample size of some studies is small, the races and age ranges of different subjects are different, and the heterogeneity of the subjects is large, which will limit the universality of the research results; for the limitations of research tools, most of the studies are completed through the subjective scale, which has a certain recall bias and cannot be monitored by objective means.

To sum up, the sleep time and sleep quality of the elderly are closely associated with their emotional and cognitive function. The worse the sleep quality is, the greater the risk of cognitive impairment is and the more serious the anxiety and depression are. Furthermore, poor mood will further aggravate the impairment of cognitive function.

## Figures and Tables

**Table 1:** Comparison of sleep quality between the two groups.

Group	Cases	PSQI	Sleep quality	Time to fall asleep	Sleeping time	Sleep efficiency
Normal cognitive function group	36	6.74 ± 2.08	1.27 ± 0.33	1.02 ± 0.73	0.78 ± 0.82	0.57 ± 0.43
Cognitive impairment group	36	8.57 ± 3.61	1.82 ± 0.64	1.43 ± 0.55	1.17 ± 0.66	1.32 ± 0.76
*t*		2.635	4.583	2.691	2.223	5.153
*P*		0.010	0.0001	0.009	0.029	0.0001

**Table 2:** Comparison of sleeping subitem scores between the two groups.

Group	Cases	Nocturnal sleep disorder	Hypnotic drug use	Daytime dysfunction	ESS score
Normal cognitive function group	36	1.14 ± 0.28	0.35 ± 0.85	1.69 ± 1.08	3.45 ± 2.61
Cognitive impairment group	36	1.67 ± 0.64	0.51 ± 1.03	1.43 ± 0.87	1.82 ± 1.47
*t*		4.552	0.719	1.125	3.265
*P*		0.0001	0.475	0.265	0.002

**Table 3:** Comparison of cognitive function between the two groups (I).

Group	Cases	MoCA	Visual space execution	Delayed recollection	Orientation
Normal cognitive function group	36	23.67 ± 1.78	4.28 ± 0.63	1.34 ± 1.08	5.83 ± 0.56
Cognitive impairment group	36	22.02 ± 3.31	3.06 ± 0.94	2.43 ± 1.56	5.74 ± 1.09
*t*		2.634	6.469	3.447	0.441
*P*		0.010	0.0001	0.001	0.661

**Table 4:** Comparison of cognitive function between the two groups (II).

Group	Cases	Naming	Attention	Language	Abstract
Normal cognitive function group	36	2.87 ± 0.23	5.34 ± 0.62	2.46 ± 0.67	1.72 ± 0.64
Cognitive impairment group	36	2.81 ± 0.52	4.49 ± 0.57	2.29 ± 0.83	1.43 ± 0.72
*t*		0.633	6.056	0.956	1.806
*P*		0.529	0.0001	0.342	0.075

**Table 5:** Comparison of anxiety and depression scores between the two groups.

Group	Cases	HAMA	HAMD
Normal cognitive function group	36	11.34 ± 6.72	5.13 ± 1.08
Cognitive impairment group	36	23.02 ± 8.75	18.63 ± 7.91
*t*		6.352	10.146
*P*		0.0001	0.0001

**Table 6:** Correlation between sleep quality, sleep time, and cognitive scale scores.

Variable	PSQI		ESS	
	*r*	*P*	*r*	*P*
MoCA	-0.487	<0.05	-0.517	<0.05
MMSE	-0.634	<0.05	-0.532	<0.05

**Table 7:** Correlation between sleep quality, sleep time, and emotional score.

Variable	PSQI		ESS		
	*r*	*P*	*r*	*P*
HAMA	0.237	<0.05	-0.416	<0.05
HAMD	0.218	<0.05	-0.387	<0.05

## Data Availability

No data were used to support this study.

## References

[1] Wesselius H. M., van den Ende E. S., Alsma J. (2018). Onderzoeks Consortium Acute Geneeskunde Acute Medicine Research Consortium. Quality and Quantity of Sleep and Factors Associated With Sleep Disturbance in Hospitalized Patients. *JAMA Internal Medicine*.

[2] Pinto J., van Zeller M., Amorim P. (2020). Sleep quality in times of Covid-19 pandemic. *Sleep Medicine*.

[3] Gao C., Chapagain N. Y., Scullin M. K. (2019). Sleep duration and sleep quality in caregivers of patients with dementia. *JAMA Network Open*.

[4] Frohnhofen H., Popp R., Stieglitz S., Netzer N., Danker-Hopfe H. (2020). Assessment of sleep and sleep disorders in geriatric patients. *Zeitschrift für Gerontologie und Geriatrie*.

[5] Rafii F., Ameri F., Haghani H., Ghobadi A. (2020). The effect of aromatherapy massage with lavender and chamomile oil on anxiety and sleep quality of patients with burns. *Burns*.

[6] Tian R., Guo Y., Luo Y. (2021). Effect of sleep quality on cognitive function in elderly hemodialysis patients. *Chinese Journal of Geriatrics*.

[7] Akinci B., Aslan G. K., Kiyan E. (2018). Sleep quality and quality of life in patients with moderate to very severe chronic obstructive pulmonary disease. *The Clinical Respiratory Journal*.

[8] Lee S. Y., Kang J. (2020). Effect of virtual reality meditation on sleep quality of intensive care unit patients: a randomised controlled trial. *Intensive & Critical Care Nursing*.

[9] Mikołajczyk-Solińska M., Śliwińska A., Kosmalski M., Drzewoski J. (2020). The phenotype of elderly patients with type 2 diabetes mellitus and poor sleep quality. *International Journal of Environmental Research and Public Health*.

[10] McDonnell B., Newcomb P. (2019). Trial of essential oils to improve sleep for patients in cardiac rehabilitation. *Journal of Alternative and Complementary Medicine*.

[11] Ansok C. B., Khalil L. S., Muh S. (2020). Objective assessment of sleep quality in patients with rotator cuff tears. *Orthopaedics & Traumatology, Surgery & Research*.

[12] Şentürk A., Tekinsoy K. P. (2018). The effect of lavender oil application via inhalation pathway on hemodialysis patients' anxiety level and sleep quality. *Holistic nursing practice*.

[13] Ramezani Kermani A., Aghebati N., Mohajer S., Ghavami V. (2020). Effect of guided imagery along with breathing relaxation on sleep quality of the elderly patients under abdominal surgery: a randomized clinical trial. *Holistic Nursing Practice*.

[14] Abdelbasset W. K., Osailan A. (2020). Sleep quality and ventilatory efficiency in elderly heart failure patients: a pilot study on the short-term effect of 4-week low-intensity aerobic exercise. *Kardiologiia*.

[15] Wang X., Lan G. (2020). Effect of targeted intervention based on subjective and objective sleep perception bias on sleep and quality of life in elderly patients with lung cancer. *Chinese Journal of Gerontology*.

[16] Yanyan F., Wanting J., Zheng X., Xing W. (2020). Meta analysis of the effect of exercise on sleep quality in elderly patients with sleep disorder. *Chinese Journal of physical Medicine and Rehabilitation*.

[17] Qin Z., Xun G., Xuanxuan W., Zheng W., Xiang Z. (2017). Sleep quality and its influencing factors in elderly patients with insomnia. *Chinese Journal of Gerontology*.

[18] Pini L., Wennberg A., Mitolo M. (2020). Quality of sleep predicts increased frontoparietal network connectivity in patients with mild cognitive impairment. *Neurobiology of Aging*.

[19] Fekih-Romdhane F., Mhedhbi N., Ben Ali S., Cheour M. (2020). Sleep quality in caregivers of older patients with schizophrenia spectrum and bipolar disorders: a case-control study. *Clinical Gerontologist*.

[20] Nobeschi L., Zangirolami-Raimundo J., Cordoni P. K. (2020). Evaluation of sleep quality and daytime somnolence in patients with chronic obstructive pulmonary disease in pulmonary rehabilitation. *BMC Pulmonary Medicine*.

[21] Xi Z., Zhengrong Y., Li Z. (2021). Effects of daily activity ability, sleep quality and their interaction on cognitive function in the elderly. *Modern preventive medicine*.

[22] Kaili Z., du Xueyun W. S. (2021). Study on neuropsychological and sleep microstructure changes in patients with circadian dysrhythmia sleep-awakening disorder with depression and anxiety treated by transcranial magnetic stimulation. *Chinese Journal of Rehabilitation Medicine*.

[23] Taishan T., Zongqiong S., Wei C., Zaohuo C., Peng Z. (2021). Magnetic resonance spectroscopy study on cognitive function and metabolites of dorsolateral prefrontal cortex in patients with chronic insomnia. *Chinese Journal of Neuropsychiatric Diseases*.

[24] Hu H., Li H., Huang X. (2020). Association of self-reported sleep duration and quality with BaPWV levels in hypertensive patients. *Hypertension Research*.

[25] Magnusdottir S., Hilmisson H. (2018). Ambulatory screening tool for sleep apnea: analyzing a single-lead electrocardiogram signal (ECG). *Sleep and Breathing*.

[26] Lu Y., Jiasi L. I., Zhou S. (2021). Correlation between somatization symptoms and BMI, sleep and cognitive function in patients with depression. *Chinese Journal of Behavioral Medicine and brain Science*.

[27] Kim J., Lee S. H., Kim T. H. (2020). Improvement of sleep quality after treatment in patients with lumbar spinal stenosis: a prospective comparative study between conservative versus surgical treatment. *Scientific Reports*.

[28] Guanghui C., Shaojie L., Qingyue K. (2021). Study on the relationship between sleep quality, depressive symptoms and their interaction with cognitive impairment in the elderly. *Chinese general practice*.

[29] Wenjing J., Peiyan S., Ma J. (2020). Study on the relationship between mild cognitive impairment and sleep disorder in the elderly. *Chinese Journal of Geriatrics*.

[30] Mahendran R., Gandhi M., Moorakonda R. B. (2018). Art therapy is associated with sustained improvement in cognitive function in the elderly with mild neurocognitive disorder: findings from a pilot randomized controlled trial for art therapy and music reminiscence activity versus usual care. *Trials*.

[31] Hogan K. J., Bratzke L. C., Hogan K. L. (2018). Informed consent and cognitive dysfunction after noncardiac surgery in the elderly. *Anesthesia and Analgesia*.

[32] Smith P. F. (2020). Why dizziness is likely to increase the risk of cognitive dysfunction and dementia in elderly adults. *The New Zealand Medical Journal*.

[33] Peng Z., Jiang H., Wang X. (2019). The efficacy of cognitive training for elderly Chinese individuals with mild cognitive impairment. *BioMed Research International*.

